The article "Analysis of the Causes and Preventive Strategies of Urogenic Sepsis after Flexible Ureteroscopic Lithotripsy" was retracted in 2023. Reasons: unreliable results or conclusions; lack of ethics approval or compliance; concerns about the data; concerns about the peer review.

# Analysis of the Causes and Preventive Strategies of Urogenic Sepsis after Flexible Ureteroscopic Lithotripsy

**DOI:** 10.1155/2022/5332101

**Published:** 2022-09-08

**Authors:** Ning Tan, Lili Xu, Jiang Wu

**Affiliations:** ^1^The Second Affiliated Hospital, Department of Urology, Hengyang Medical School, University of South China, Hengyang 421001, Hunan, China; ^2^The Second Affiliated Hospital, Department of Oncology Hematology, Hengyang Medical School, University of South China, Hengyang 421001, Hunan, China; ^3^The Second Affiliated Hospital, Department of General Surgery, Hengyang Medical School, University of South China, Hengyang 421001, Hunan, China

## Abstract

**Objective:**

To explore the causes of urogenic sepsis in patients after flexible ureteroscopic lithotripsy and analyze the preventive strategies.

**Methods:**

A total of 240 patients who underwent flexible ureteroscopic lithotripsy in our hospital from January 2019 to June 2022 were selected and divided into 2 groups according to whether postoperative ureteral sepsis occurred. 24 cases occurred in the observation group. Logistics multivariate regression analysis was used to analyze the risk factors of urogenic sepsis after flexible ureteroscopic lithotripsy, and the serum albumin (ALB), the peripheral blood neutrophil-to-lymphocyte ratio (NLR), and the level of procalcitonin (PCT) were correlated, and the ROC curve was used to analyze the predictive value of each index for urosepsis.

**Results:**

Univariate analysis showed that there were differences in gender, age, diabetes, stone diameter, and urine culture ratio between the two groups (*P* < 0.05). The results of multivariate regression analysis showed that female, age ≥60 years, stone diameter >2.5 cm, and positive urine culture were the main influencing factors for the occurrence of urogenic sepsis. After operation, the ALB levels in the two groups were lower than those before operation, and the levels of NLR and PCT in the two groups were higher than those before operation; the ALB levels in the observation group were lower than those in the control group, and the NLR and PCT in the observation group were higher than those in the control group (*P* < 0.05). According to Spearman's correlation analysis, ALB was negatively correlated with the occurrence of uremia (*P* < 0.05), *r* = −0.320, NLR and PCT were positively correlated with the occurrence of uremia (*P* < 0.05), *r* = 0.313, respectively, and 0.417; in addition, Pearson's correlation analysis showed that ALB was negatively correlated with NLR and PCT in the two groups (*P* < 0.05, *r* = −0.507, −0.605 in the control group, respectively, and *r* were −0.452 and −0.412 in the observation group). There was a positive correlation between NLR and PCT (*P* < 0.05), *r* = 0.840, and there was no correlation between NLR and PCT in the observation group (*P* > 0.05). According to the ROC curve analysis, the predictive value AUC of ALB, NLR, PCT and combined use were 0.808, 0.801, 0.901, and 0.925 (*P* < 0.05).

The article "Analysis of the Causes and Preventive Strategies of Urogenic Sepsis after Flexible Ureteroscopic Lithotripsy" was retracted in 2023. Reasons: unreliable results or conclusions; lack of ethics approval or compliance; concerns about the data; concerns about the peer review.

**Conclusion:**

Gender, age, stone diameter, and urine culture results are the main influencing factors for the occurrence of urinary sepsis. Therefore, preventive measures should be strengthened for this group of patients. In addition, the combined use of postoperative ALT, NLR, and PCT level tests can be better.

## 1. Introduction

Urinary calculi is a relatively common urological disease with a high incidence rate, and with the change of people's living environment and lifestyle, the incidence rate is on the rise [1, 2]. In addition, urinary calculi can cause acute or chronic pain in patients and lead to symptoms such as hematuria and infection, which seriously endanger the health of patients and increase their physical and life burden [3]. Currently, patients with urinary calculi are mostly treated with endoscopic surgery. Among them, ureteroscopic surgery has the advantages of a clear surgical field, small incision, and quick postoperative recovery, and has become one of the more widely used surgical methods [4, 5]. Although the effect of ureteroscopic surgery is good, postoperative complications cannot be avoided. Among the complications, the incidence of postoperative infection is the highest. Urinary-derived infection is a high risk of postoperative infection, which has a rapid onset and can lead to systemic inflammatory response syndrome in patients, with high mortality and high harm to patients [6]. Early identification of postoperative urosepsis and early intervention can improve the prognosis of patients. Therefore, it is of great significance to find urosepsis markers with good sensitivity and rapid detection. Serum albumin (ALB) is a sensitive nutritional marker, and studies have shown that it can predict the prognosis of patients undergoing surgical treatment, and peripheral blood neutrophil-to-lymphocyte ratio (NLR) can reflect the immune status of patients. Procalcitonin (PCT) is an infection-related factor, which can be used to diagnose sepsis [7–9]. Therefore, this study investigated the causes of urogenic sepsis in patients after flexible ureteroscopic lithotripsy and analyzed the predictive value of ALB, NLR, and PCT for postoperative urogenic sepsis so as to provide an effective basis for preventive strategies.

## 2. Materials and Methods

### 2.1. General Information

A total of 240 patients who underwent flexible ureteroscopic lithotripsy in our hospital from January 2019 to June 2021 were selected, including 112 males and 128 females, aged 20–76 years, with an average of (54.90 ± 12.26) years old, and 122 patients with diabetes mellitus. For example, the stone diameter was (2.34 ± 0.97) cm. They were divided into 2 groups according to the occurrence of postoperative urinary sepsis. The diagnostic criteria were referred to as the “China Emergency Treatment Guidelines for Severe Sepsis/Septic Shock (2018)” [10]. 24 cases occurred in the observation group. This study was carried out with the approval of the Ethics Committee of The Second Affiliated Hospital, Hengyang Medical School, and University of South China (2018010).

The article "Analysis of the Causes and Preventive Strategies of Urogenic Sepsis after Flexible Ureteroscopic Lithotripsy" was retracted in 2023. Reasons: unreliable results or conclusions; lack of ethics approval or compliance; concerns about the data; concerns about the peer review.

### 2.2. Inclusion Criteria

①All patients are >18 years old; ② Informed consent of patients and their families; ③ the patient's treatment compliance is good; ④ the patient was diagnosed with ureteral calculi by preoperative imaging test; ⑤ the patient's clinical data are complete.

### 2.3. Exclusion Criteria

① Patients with malignant tumor; ② those who suffer from mental illness or cannot communicate normally; ③ suffering from other cardiovascular and cerebrovascular diseases; ④ suffering from infectious diseases; ⑤ those who are pregnant or breastfeeding; ⑥ combined with other urinary system diseases.

### 2.4. Methods

#### 2.4.1. Preoperative

Routine examinations, serum biochemical examinations, and urine culture examinations were performed on all patients upon admission. Routine examinations include imaging examinations such as B-ultrasound and CT. At the same time, in order to accurately assess the patient's physical condition, other targeted examination items are expanded according to the actual situation of the patient.

#### 2.4.2. Serum Biochemical Test

Instruct the patient to fast the night before, and drink a small amount of water. In the early morning of the second day, blood is drawn from the peripheral cubital vein of the patient in fasting state, and 5 mL of blood is drawn, which is divided into two test tubes for use, and one tube was used to measure serum albumin (ALB) and procalcitonin (PCT) levels, and the other was used to measure peripheral blood neutrophil-to-lymphocyte ratio (NLR).

#### 2.4.3. Urine culture

For male patients, the foreskin is turned up during urination to collect urine; for female patients, first wash the patient's vulva with soapy water, and then wash with normal saline for a second time, and use the method of separating the labia when urinating so as to collect urine; the urination process was not interrupted, and the urine was sent for examination immediately after collection. If the urine culture is positive, antibiotics should be given before surgery, and a second examination should be performed. The urine culture result was negative before surgery.

The article "Analysis of the Causes and Preventive Strategies of Urogenic Sepsis after Flexible Ureteroscopic Lithotripsy" was retracted in 2023. Reasons: unreliable results or conclusions; lack of ethics approval or compliance; concerns about the data; concerns about the peer review.

#### 2.4.4. Intraoperative

All patients were under general anesthesia, and in order to ensure a clear field of vision during the operation, they were irrigated with normal saline. Then, the thickness and dilatation ability of the patient's ureter were checked with a rigid ureteroscope. After the confirmation, a zebra guide wire was inserted into the ureter at the opening of the patient's ureteral calculi. Immediately, the ureteroscope was expanded along the zebra guide wire to determine the position of the patient's stone. After a stone is found, a lithotripsy operation is performed using a holmium laser. After the lithotripsy was completed, the ureteroscope was taken out, the zebra guide wire was indwelled, and the F6 double J tube was indwelled by the zebra guide wire.

### 2.5. Observation Indicators

The patients were examined upon admission, and their clinical data were collected and sorted, including gender, age, diabetes, and BMI.

ALB, NLR, and PCT were measured before and after surgery, and urine culture results were recorded. The patient's neutrophils and lymphocytes were detected by an automatic blood analyzer (Shanghai Huanxi Medical Instrument Co., Ltd., model BC-5180). ALB and PCT were detected by the Elisa kit (Shanghai Enzyme Link Biotechnology Co., Ltd.). The operation time and stone diameter of the patients were recorded after the operation.

### 2.6. Statistical Methods

The SPSS21.0 statistical software was used for data analysis, measurement data were expressed as ($\bar{x}$ ±*s*), *t*-test was used, count data was expressed as %, 2 test was used, and logistic regression analysis was used to analyze the effect of urosepsis Factors were analyzed, Spearman and Pearson methods were used for correlation analysis, and the ROC curve was used to analyze the predictive value. When *P* < 0.05, the difference was statistically significant.

## 3. Results

### 3.1. Univariate Analysis Results

A total of 240 cases were included in this study, of which 216 cases did not develop urosepsis, and 24 cases developed urosepsis, and univariate analysis was performed. The results showed that there were significant differences in gender, age, diabetes, stone diameter and urine culture ratio between the two groups (*P* < 0.05) as shown in Table 1.

### 3.2. Results of Multivariate Analysis

Taking the occurrence of urogenic sepsis as the dependent variable, assign the value. No urogenic sepsis is 0, and 1 is the occurrence of urogenic sepsis. Gender, age, diabetes mellitus, stone diameter, and urine culture were used as covariates to assign values, male was 0, female was 1, age <60 years was 0, age >60 years was 1, and no diabetes was 0, 1 for diabetes, 0 for stone diameter ≤2.5 cm, 1 for stone diameter >2.5 cm, 0 for negative urine culture, 1 for positive urine culture, multivariate regression analysis was performed. The results of multivariate regression analysis showed that females, age ≥60 years, stone diameter >2.5 cm and positive urine culture were the main influencing factors for the occurrence of urogenic sepsis as shown in Table 2.

The article "Analysis of the Causes and Preventive Strategies of Urogenic Sepsis after Flexible Ureteroscopic Lithotripsy" was retracted in 2023. Reasons: unreliable results or conclusions; lack of ethics approval or compliance; concerns about the data; concerns about the peer review.

### 3.3. Comparison of Postoperative ALB, NLR, and PCT Levels between the Two Groups of Patients

There was no significant difference in the levels of ALB, NLR, and PCT between the two groups before surgery (*P* > 0.05). The levels of ALB in the two groups after operation were lower than those before operation, the levels of NLR and PCT in the two groups were higher than those before operation, and the level of ALB in the observation group was lower than that in the control group. The NLR and PCT in the observation group were higher than those in the control group, and the difference was statistically significant (*P* < 0.05). As shown in Table 3.

### 3.4. Correlation Analysis Results

Correlation analysis was performed using Spearman's method. The results showed that ALB was negatively correlated with the occurrence of urosepsis (*P* < 0.05), *r* = −0.320, and NLR and PCT were positively correlated with the occurrence of urosepsis (*P* < 0.05), and *r* was 0.313 and 0.417. In addition, Pearson's method was used to analyze the correlation of each index. The results showed that ALB was negatively correlated with NLR and PCT in the two groups (*P* < 0.05, *r* was −0.507 and −0.605 in the control group, and *r* was −0.452 and −0.412 in the observation group, respectively), and the control group was positively correlated with NLR and PCT (*P* < 0.05), *r* = 0.840, There was no correlation between NLR and PCT in the observation group (*P* > 0.05) as shown inTables 4–6 and Figures 1 and 2.

### 3.5. The Predictive Value of ALB, NLR, and PCT for Ureteral Sepsis after Flexible Ureteroscopic Lithotripsy

Taking the occurrence of urogenic sepsis as the dependent variable, assigning value, no urogenic sepsis is 0, the occurrence of urogenic sepsis is 1, and ROC curve analysis is performed. The results showed that the ALB, NLR, PCT and combined use predicted value AUC were 0.808, 0.801, 0.901 and 0.925, respectively. It was statistically significant (*P* < 0.05) as shown in Table 7 and Figure 3.

## 4. Discussions

Urinary sepsis is one of the critical illnesses. It is a sepsis caused by urinary system infection, which can cause a systemic inflammatory response, and the mortality rate is as high as 35%–75%, which seriously endangers the life safety of patients [11, 12]. With the widespread application of endoscopic lithotripsy, postoperative ureteral sepsis has occurred frequently, and the incidence of ureteral sepsis after ureteroscopic surgery is about 4.5% [13]. Therefore, early detection and targeted treatment are of great significance to the prognosis of patients.

The article "Analysis of the Causes and Preventive Strategies of Urogenic Sepsis after Flexible Ureteroscopic Lithotripsy" was retracted in 2023. Reasons: unreliable results or conclusions; lack of ethics approval or compliance; concerns about the data; concerns about the peer review.

Urinary sepsis is caused by urinary system infection, and PCT is closely related to infection. Due to infection, the toxin content in the body is too high, and the PCT in the body increases, reaches a high level within 12–48 hours, and it has good stability, so it has high value for the diagnosis of infectious diseases [8]. However, it takes a certain period of time for the level of PCT to increase, which causes a certain delay in the early diagnosis of urosepsis. Secondly, NLR can reflect the patient's immune status. When the patient develops urosepsis, it will trigger a systemic inflammatory response, a large number of T lymphocytes will be depleted, and the immune system will be disturbed. Neutrophils fail to reach the infection site, and NLR will follow the rise. In addition, sepsis will promote the increase of capillary permeability in patients, resulting in a decrease in ALB levels, hypoalbuminemia, and rapid changes in ALB levels, so the risk of disease can be predicted based on ALB levels. However, it should be noted that ALB will decrease after surgery and when the body responds to stress, so there is a certain error in the prediction of a single index.

The results of this study showed that univariate analysis showed that there were differences in gender, age, diabetes, stone diameter, and urine culture ratio between the two groups. Diameter >2.5 cm and positive urine culture are the main influencing factors for the occurrence of urogenic sepsis. Analysis of the reasons: female is the main factor may be that the urethral opening is close to the vaginal opening and anus, thereby increasing the risk of infection, similar to other [2] studies. Secondly, due to the gradual decline of physical functions, elderly patients have poor resistance to infection and a higher risk of disease. In addition, if the patient's stone diameter is too large, there will be more bacteria in the stone, and during the intraoperative lithotripsy operation, more fragments will be generated, which will lead to a longer treatment time and increase the risk of infection. On the other hand, the preoperative urine culture was positive. Although the secondary urine culture was negative after antibiotic treatment, the operation was performed, but most of the stones contained bacterial endotoxins, and it was difficult for antibiotics to enter the stones. During lithotripsy, large amounts of endotoxins are released into the body, increasing the risk of infection. In addition, the levels of ALB in the two groups after surgery were lower than those before surgery, and the levels of NLR and PCT in the two groups were higher than those before surgery, and the levels of ALB in the observation group were lower than those in the control group, and the NLR and PCT in the observation group were higher than those in the control group, indicating that ALB in the urine. In patients with primary sepsis, due to the increased capillary permeability of the body, the level of decline is even greater, so the risk of disease can be predicted to a certain extent, and patients with sepsis develop systemic inflammatory responses due to infection and immune system disorders, resulting in increased NLR levels in patients, while PCT also increased due to infection. At the same time, ALB was negatively correlated with the occurrence of urosepsis, NLR and PCT were positively correlated with the occurrence of urosepsis, ALB was negatively correlated with NLR and PCT in the two groups, and NLR and PCT were positively correlated in the control group, indicating that each index has a certain synergistic effect in predicting urogenic sepsis, similar to other studies [14]. However, there was no correlation between NLR and PCT in the observation group in this study, and the reason for the analysis may be that there were fewer cases, which led to deviations in the results. After ROC curve analysis, the combined multi-index diagnosis AUC is the largest, indicating the highest predictive value. Therefore, attention should be paid to patients with lower levels of ALB and higher levels of NLR and PCT after surgery, and they should always be ready to detect various vital signs of patients.

The article "Analysis of the Causes and Preventive Strategies of Urogenic Sepsis after Flexible Ureteroscopic Lithotripsy" was retracted in 2023. Reasons: unreliable results or conclusions; lack of ethics approval or compliance; concerns about the data; concerns about the peer review.

In conclusion, gender, age, stone diameter, and urine culture results are the main influencing factors for the occurrence of urogenic sepsis. Therefore, for such groups, preventive measures should be strengthened. In addition, postoperative ALT, NLR, and PCT levels can better predict whether the patient will develop urosepsis so it can be detected early and targeted treatment can be started as soon as possible. There are still shortcomings in this study; the selected cases are small, the results may be biased, and no in-depth investigation of patient prognosis has been carried out, and the next study will further follow up.

## Figures and Tables

**Figure 1:** Scatter plot between each index in the control group.

**Figure 2:** Scatter plot between each index in the observation group.

**Figure 3:** ROC chart of the predictive value of ALB, NLR, and PCT for ureteral sepsis after flexible ureteroscopic lithotripsy.

**Table 1:** Results of univariate analysis.

Indexes		Control group (*n* ＝ 216)	Observation group (*n* ＝ 24)	*χ* ^*2*^/*t*	*P*
Gender	Male	106	6	5.030	0.025
	Female	110	18		

Age	<60 year	120	8	4.286	0.038
	≥60 year	96	16		

Whether have diabetes	Yes	105	17	4.268	0.039
	No	111	7		

Operation time		46.24 ± 12.17	50.45 ± 15.93	1.524	0.129

Stone diameter	≤2.5 cm	137	10	4.309	0.038
	>2.5 cm	79	14		

Urine culture	Positive	57	11	4.022	0.045
	Negative	159	13		

BMI (kg/m^2^)		26.21 ± 4.52	26.48 ± 3.75	0.282	0.778

**Table 2:** Results of multivariate analysis.

Influencing factors	*β* value	Se value	Wald value	*P* value	OR value	95%CI
Gender	1.339	0.524	6.522	0.011	3.815	(1.365, 10.659)
Age	0.979	0.475	4.237	0.040	2.661	(1.048, 6.755)
Stone diameter	1.280	0.476	7.231	0.007	3.598	(1.415, 9.147)
Urine culture	1.095	0.469	5.466	0.019	2.990	(1.194, 7.491)
Constant	−4.604	0.718	41.103	0.001	0.010	

**Table 3:** Comparison of postoperative ALB, NLR, and PCT levels in two groups of patients.

Group	ALB (g/L)		NLR		PCT (ng/mL)	
	Preoperative	Postoperative	Preoperative	Postoperative	Preoperative	Postoperative
Control group (*n* = 216)	39.44 ± 2.73	37.15 ± 3.54^①^	4.78 ± 1.95	5.25 ± 1.31^①^	1.26 ± 0.33	1.38 ± 0.27^①^
Observation group (*n* = 24)	38.72 ± 2.16	33.24 ± 2.87^①^	4.53 ± 1.66	7.24 ± 1.96^①^	1.31 ± 0.25	2.74 ± 1.01^①^
*t*	1.249	5.221	0.604	6.672	0.719	15.587
*P*	0.213	<0.001	0.546	<0.001	0.473	<0.001

Note. Compared with before operation, ^①^*P* < 0.05.

**Table 4:** The results of correlation analysis between each index and the occurrence of urosepsis.

Indexes	Whether urosepsis occurs	
	*r*	*P*
ALB	−0.320	<0.001
NLR	0.313	<0.001
PCT	0.417	<0.001

**Table 5:** The results of the correlation analysis between the indicators in the control group.

Indexes	ALB		NLR		PCT	
	*r*	*P*	*r*	*P*	*r*	*P*
ALB	—	—	−0.507	<0.001	−0.605	<0.001
NLR	−0.507	<0.001	—	—	0.840	<0.001
PCT	−0.605	<0.001	0.840	<0.001	—	—

**Table 6:** Correlation analysis between each index in the observation group.

Indexes	ALB		NLR		PCT	
	*r*	*P*	*r*	*P*	*r*	*P*
ALB	—	—	−0.452	0.027	−0.412	0.045
NLR	−0.452	0.027	—	—	0.324	0.123
PCT	−0.412	0.045	0.324	0.123	—	—

**Table 7:** The predictive value of ALB, NLR, and PCT for ureteral sepsis after flexible ureteroscopic lithotripsy.

Indexes	AUC	*P*	95%CI	Sensitivity	Specificity
ALB	0.808	<0.001	(0.725, 0.891)	0.750	0.759
NLR	0.801	<0.001	(0.691, 0.911)	0.667	0.870
PCT	0.901	<0.001	(0.799, 1.000)	0.833	0.968
Joint	0.925	<0.001	(0.841, 1.000)	0.875	0.935

The article "Analysis of the Causes and Preventive Strategies of Urogenic Sepsis after Flexible Ureteroscopic Lithotripsy" was retracted in 2023. Reasons: unreliable results or conclusions; lack of ethics approval or compliance; concerns about the data; concerns about the peer review.

## Data Availability

The data can be obtained from the author upon reasonable request.
